This article has been retracted.

# Influence of Virtual Reality Technology on Clinical Thinking Cultivation of Medical Students

**DOI:** 10.1155/2021/8004883

**Published:** 2021-08-12

**Authors:** Yuying Wang

**Affiliations:** ^1^College of Information Science and Technology, Northeast Normal University, Changchun, China; ^2^Modern Education Technology Center, Jilin Medical University, Jilin, China

## Abstract

Clinical thinking is not only the basis and premise of clinical reasoning and decision-making, but the necessary quality to cultivate reliable, responsible, and emotional excellent doctors. Virtual reality technology provides a real clinical learning environment for medical students, which can bridge the gap between medical theory and medical practice and save educational resources. Virtual reality is helpful to cultivate medical students' clinical thinking and prepare for their clinical practice. Through the deconstruction of clinical thinking, this paper determines the connotation and constituent elements of clinical thinking, puts forward the model framework for virtual reality technology to promote the development of medical students' clinical thinking, and explains the impact of virtual reality technology on the development of medical students' clinical thinking, clinical reasoning, and critical thinking from the aspects of virtual reality situation, teaching activities, and virtual reality characteristics.

## 1. Introduction

### 1.1. Clinical Thinking Cultivation Is the Demand of Medical Talent Training

China puts forward the implementation of healthy China strategy, establishes the concept of “great health,” deepens the cooperation between medicine and education, promotes the competency-oriented education and teaching reform, optimizes the medical professional structure serving the whole life cycle and the whole process of health, promotes the deep integration of information technology and medical education, cultivates first-class medical talents, and serves the construction of healthy China [1–3]. To meet the requirements of the construction of “new medicine” in China, we should take learners as the center, reshape new forms of education and teaching, and promote the application of new generation of information technology such as virtual reality in medical education [4]. Under the background of healthy China construction strategy and the rapid development of information and digital technology, virtual reality will become an indispensable teaching and training means in the medical industry and will play a more extensive role in the training of new medical talents and clinical thinking of medical students [5, 6]. It is necessary to continuously promote the competency-oriented education and teaching reform and strive to improve the clinical practice ability of medical students. Clinical practice teaching is an important link to complete the cultivation of clinical thinking, skills, and practical clinical work ability of medical students. However, medical students lack the opportunity to contact patients for clinical practice in the clinical learning stage, which hinders the cultivation of medical students. Therefore, in order to improve this situation as soon as possible, integrating medical teaching resources, cultivating medical students' clinical thinking, and introducing virtual reality technology into medical teaching can effectively solve many problems in medical personnel cultivation [7, 8]. In the process of cultivating medical students' clinical thinking, we should make use of the deep integration of information technology and disciplines to cultivate modern innovative medical talents and serve the construction of healthy China.

### 1.2. Problems in the Cultivation of Clinical Thinking

There are many problems in the process of clinical thinking training. The cultivation of clinical thinking ability of medical students in many colleges and universities is an important part of teaching reform, but it does not really reflect the hierarchical cultivation of clinical thinking ability in practical education. Students are passive in the process of clinical practice and under the guidance of teachers in clinical practice, and they have less opinion when dealing with cases, which affects the effect of teaching. Some students do not pay enough attention to clinical thinking ability. They think that as long as they master enough advanced equipment and instruments, they can effectively diagnose and treat diseases, which has an impact on the cultivation of clinical thinking ability. In clinical practice, there are limited cases, trial and error are not allowed, and the teaching level is not consistent with that of clinicians and clinical nurses, which makes it difficult for students to change their thinking. The low utilization rate of high-end teaching equipment also limits the use frequency of students and affects the quality of medical practice teaching. However, there are some disadvantages in medical experiment teaching, such as high cost, high risk, and irreversibility [9–11].

### 1.3. Virtual Reality Technology Provides a Good Support for the Development of Clinical Thinking

Using virtual reality technology to provide students with a practical clinical learning environment can cultivate medical students' clinical thinking and improve their clinical practice preparation ability. The simulation project based on virtual reality technology guides students to comprehensively use multidisciplinary knowledge to solve clinical problems of patients in different scenes, aiming to improve their clinical thinking ability of finding and solving problems [12]. The virtual simulation experiment teaching project creates a real situation close to the clinical situation, so that students can quickly adapt to complex clinical scenes by understanding and applying the theoretical knowledge they have learned. In order to better solve the practical problems of patients and clinical practical problems, we should construct our own knowledge system, organically combine theory with practice, and promote the development of clinical thinking, so as to promote professional growth [13]. Virtual reality has many advantages in the cultivation of clinical thinking. It can avoid risks, make up for many shortcomings in modern medical teaching, and save educational resources. The practical application is not limited by time and space and improves the teaching efficiency. Situational teaching and interaction can be carried out to stimulate students' learning enthusiasm and innovation, which is conducive to cultivating innovative consciousness and clinical thinking [14].

## 2. Research on Clinical Thinking

### 2.1. Meaning of Clinical Thinking

The concept of clinical thinking has not been unified. Bordage believes that the clinical knowledge stored in the brain of clinicians and the flexibility of their thinking enable them to accurately and efficiently carry out clinical reasoning and diagnosis. Clinical reasoning is an important practical way of clinical thinking [15]. Likhterman et al. define clinical thinking as the ability of doctors to cover, analyze, and synthesize all available data and information of patients, acquire relevant knowledge and intuition from books, and formulate diagnosis, prognosis, and treatment strategies [16]. Chris et al. believe that clinical thinking is a process of logical analysis in daily work to find, analyze, and solve problems from different perspectives. They analyzed how doctors and experts make key decisions. Experts seem to use their intuition or experience to match each new situation with existing cases and plans and use the existing cases and plans to decide an action plan [17]. Fuks et al. believe that clinical thinking is the whole cognitive process of health professionals in the process of work. It includes clinical inquiry, clinical reasoning, and clinical judgment [18]. Wang thinks that clinical thinking is the diagnostic thinking and therapeutic thinking of medical staff in clinical practice on the diagnosis, treatment, prognosis, and prevention of diseases [19].

Zeng and Lu pointed out that clinical thinking refers to the use of medical, natural science, humanities and social sciences and behavioral science knowledge, taking patients as the center, combined with the best available evidence and information, and carrying out critical analysis, synthesis, analogy, judgment and differential diagnosis according to the information of patients symptoms, so as to finally form a personalized scheme of diagnosis and treatment [20]. Faucher points out that clinical thinking includes knowledge and other personal (abilities, values, ethical principles, etc.) and external (colleagues and assistants, reference materials, instruments, etc.) resources, as well as critical thinking. These are considered as the inputs of clinical reasoning, which is the core of clinical thinking. Critical thinking promotes clinical reasoning [21]. Luis thinks that clinical thinking is a very complex process, which can be described by the dual process theory. It has an intuitive part (recognition pattern) and an analytical part (hypothesis testing). It is vulnerable to cognitive biases that professionals must be aware of in order to minimize errors in diagnosis and decision-making [22]. Takata et al. pointed out that group discussion is based on the patient's medical history, history, physical examination, and laboratory data information. The data information is collected and discussed to extract meaningful problems and concepts for diagnosis, management, and decision-making. These concepts are roughly defined as clinical thinking [23]. Clinical thinking is a kind of reasoning and thinking method that doctors or medical students use with the knowledge of natural science, humanities and social science, and behavioral science to recognize and judge diseases. It is the key ability of effective clinical diagnosis and treatment. Clinical thinking starts from a complex clinical situation, which leads to the need for clinical reasoning. It also involves personal and professional judgment, so as to take wise action for each specific case. The clinical decision-making of building a harmonious and healthy doctor-patient relationship should be patient-centered, creatively and critically acquiring relevant knowledge and skills and integrating multidisciplinary professional knowledge to solve clinical problems. In this process, we should think critically about our clinical thinking ability of reasoning, judgment, and decision-making.

### 2.2. Elements of Clinical Thinking

Neistadt proposed the concept of clinical reasoning, which can be regarded as the description or thinking framework of psychological operation, a structure to organize and support clinical thinking [24]. According to Faucher, clinical thinking includes knowledge, other personal and external resources, clinical reasoning, and critical thinking. Knowledge and other personal and external resources are considered as the input of clinical reasoning. Clinical reasoning is the core of clinical thinking, and critical thinking is the promoting factor of clinical reasoning [21]. According to Faucher's definition of clinical thinking, the main elements of clinical thinking include clinical reasoning, clinical judgment, decision-making, and critical thinking. The elements of clinical thinking are shown in Figure 1.

#### 2.2.1. Clinical Reasoning

Elstein et al. believe that clinical reasoning means solving problems and making decisions [25]. Clinical reasoning is a thinking and decision-making process related to clinical practice. The cognitive process is needed to evaluate and deal with clinical problems. In the process of solving clinical problems, correct, accurate, and scientific clinical reasoning, clinical judgment, and decision-making play an important role. It teaches medical students to learn to study and think independently and plays an important role in the development of clinical thinking.

#### 2.2.2. Clinical Judgment

Clinical judgment is a general judgment made by doctors or medical students according to the history and background of patients, as well as their own professional knowledge, to examine the state of human health and the disease of patients. It is used to determine the nature of the disease, and based on this judgment, we can get correct, appropriate, and scientific treatment and prognosis through clinical reasoning. In the face of more complex medical professional practice, we need to pay special attention to a higher level of understanding, identification, judgment, and evaluation [26, 27].

#### 2.2.3. Decision Making

Decision-making is a process of thinking and decision-making related to clinical practice. Doctors diagnose patients according to relevant resources and choose the most suitable, scientific, and accurate treatment scheme for patients from a variety of treatment schemes. Clinical decision-making is also a necessary cognitive process for evaluating and managing patient-related clinical problems [28].

#### 2.2.4. Critical Thinking

As a promoting factor of clinical reasoning, critical thinking actively and skillfully analyzes the structural elements contained in clinical thinking. Critical thinking is the most basic and creative form of thinking in people's activities of understanding the world, especially in the process of reasoning, judgment, and evaluation [29]. Critical thinking is one of the driving forces to promote social progress, and its core is evaluation and judgment. Cultivating critical thinking of medical students is the key to knowledge innovation and cultivating excellent medical talents.

### 2.3. Influencing Factors of Clinical Thinking

As an open system in humans, clinical thinking not only has complex interaction between systems but also keeps close contact with the external environment. That is to say, in the process of development, clinical thinking is not only affected by system elements and external environment but also by its own characteristics. In the study of thinking structure, we should consider not only the cognitive factors of thinking but also the noncognitive factors of thinking. Similarly, as an advanced cognitive activity, clinical thinking is not only restricted by its own level, characteristics, quality, and other cognitive factors but also by its own motivation, interest, emotion, will, personality, and other noncognitive factors [30, 31]. Situational simulation teaching can promote the development of clinical thinking. Situational simulation teaching is to solve clinical problems in cases through practical cultivation, discussion, and reflection. In order to ensure the continuity and scientificity of the whole situation simulation learning, teachers should focus on guiding reflection to students after the situation simulation, which is helpful to students' meaningful learning [32]. As the core part of clinical practice ability, clinical thinking is an important part of doctors' clinical competency. Jing et al. pointed out that good clinical thinking ability is inseparable from three influencing factors: systematic theoretical knowledge, scientific thinking method, and continuous clinical practice [33]. Previous studies have shown that problem-based learning (PBL) can promote the development of clinical thinking. It is to strengthen students' ability of autonomous learning and solving practical problems by adopting the group discussion teaching method based on clinical practical problems, with students as the main body and teachers as the guidance. Jauhiainen et al. pointed out that the PBL teaching method can develop information literacy skills, critical thinking and evidence-based nursing skills, communication, cooperation, and teamwork skills, and problem-solving and self-assessment skills [34]. Learners' reflection can promote the development of clinical thinking. Reflective diary is a kind of teaching strategy often used in clinical education to understand students' clinical thinking [35].

## 3. Potential Power of Virtual Reality Technology to Promote the Development of Clinical Thinking of Medical Students

### 3.1. Theoretical Basis of Virtual Reality Technology Supporting the Cultivation of Clinical Thinking of Medical Students

Virtual reality technology to promote the development of clinical thinking of medical students is in line with the view of educational theory. Behaviorism believes that learning is a stimulus response (S-R) connection formula, and learning is completed by response from stimulation [36]. Constructivism believes that “moving the laboratory to the classroom” makes learning a real situational experience. Constructivist learning theory holds that learning is a process in which learners gradually understand the external world. On the basis of learners' existing cognitive structure and under a certain social situation, learners constantly acquire new knowledge through communication with the outside world, assimilate and adapt to their original knowledge structure, and finally achieve a balance [37]. Embodied cognition theory holds that only when learners' cognition, body, and environment interact effectively can they learn [38]. Action affects perception, which in turn affects future action, which in turn determines new perception, thus forming a “perception action cycle” [39]. Students' meaningful learning is to transfer knowledge to different situations on the premise of deep understanding of knowledge and cultivate their thinking and problem-solving ability in the form of practice or experiment. Learning under the guidance of embodied cognition theory is embodied and situational, emphasizing the influence of body and its experience on learning [40]. In order to stimulate the enthusiasm of students and improve their clinical thinking ability of reasoning, judgment, and decision-making, the simulation experiment project based on virtual reality technology is used to guide students to comprehensively use multidisciplinary knowledge to solve the clinical problems of patients in different scenes.

### 3.2. Internal Logical Relationship between Virtual Reality Technology and Clinical Thinking

Virtual reality has the characteristics of immersion, interaction, and imagination. The performance of immersive learning is that learners, as a part of the virtual reality learning environment, can more realistically feel the reality of being a participant in the virtual reality learning environment. Interaction is an efficient and natural human-computer interaction through software and hardware. It is the interaction between learners and learning environment, learning resources, learning content, and so on. Imagination is a thinking process of representation, criticism, and creation. In the virtual reality learning environment, learners can make reasoning and logical judgment according to various kinds of information in the environment and their own behavior, so as to obtain more knowledge and understand more complex deep mechanism [41, 42]. The immersion and interaction of virtual reality provide experience support for the cultivation of medical students' clinical thinking and promote the generation of learners' experience and the development of clinical thinking. Immersion and imagination provide visual spatial perception support for the cultivation of medical students' clinical thinking and promote the combination of medical theory and practice [43, 44]. Virtual reality technology promotes the cultivation of clinical thinking of medical students, as shown in Table 1.

## 4. Model Framework of Virtual Reality Technology Promoting the Development of Clinical Thinking of Medical Students

Based on the above interpretation and relationship between clinical thinking and virtual reality, this study proposes a model framework of virtual reality technology promoting the development of clinical thinking in medicine, including the methods and paths of the combination of virtual reality technology and clinical thinking. The model framework is shown in Figure 2.

### 4.1. Virtual Reality Provides Realistic Virtual Situations

We use virtual reality technology to construct real situations and enhance teachers' teaching and learners' enthusiasm and efficiency in learning. The learners' deeper learning motivation is induced and the learners' active participation and collaborative inquiry are encouraged, which is conducive to their creative completion of their knowledge construction [45]. Questions from real situations are meaningful to learners. For the traditional classroom situation, there are some problems, such as lack of authenticity and simplification. Through virtual reality technology, we can create a more real learning situation and set appropriate learning difficulties to promote learners' meaningful learning. In the learning situation created by virtual reality technology, learners reasonably analyze the situation problems, use their original knowledge to explore the situation problems, constantly approach the key and core of the problem, and make assumptions, reasoning, and judgment on the possible solutions. Learners match the available information and situation with their original cognition according to their own experience and background knowledge and use their original cognitive structure to determine the next action plan. If it can be identified and matched, clinical judgment and decision-making can be made directly. If it cannot match the original cognitive structure, it needs to deeply process the information, clarify the problems encountered, solve the problems, and reflect. The application of virtual reality technology in the understanding of medical theory, the mastery of practical skills, and the cultivation of clinical thinking has a significant effect. For example, the application of virtual reality technology in anatomy teaching can vividly and stereoscopically show its complex and abstract anatomical structure. This allows students to dissect it repeatedly, which makes up for the scarcity of teaching resources of real human specimens and also makes the anatomical theory, concept, and structure become concrete, intuitive, immersive, interactive, and three-dimensional. Researchers explore the application of virtual reality technology to clinical thinking cultivation more, and different scholars at home and abroad from different angles have proved that virtual reality technology can promote the development of clinical thinking. The results of the existing research show that virtual reality technology is a more effective learning environment in classroom than traditional teaching and has a wide application prospect. Therefore, it is necessary to pay attention to the application of virtual reality technology in clinical thinking cultivation in medicine and enrich the relevant research in the virtual reality learning environment, so as to provide more support for promoting the development of clinical thinking of medical students.

### 4.2. Teaching Activities Focusing on the Development of Clinical Thinking

Virtual reality provides massive resources and contexts for learners' deeper learning through computer technology. Teachers need to list the framework of teaching content through the knowledge integration of different modules according to different teaching goals and requirements. This is conducive to learners to assimilate the original cognitive structure with the new situation in the virtual reality learning environment to achieve meaningful learning. Virtual reality provides experience, context, and emotional support in the learning process of learners and helps learners to construct and transfer knowledge in virtual situations [46]. Jenson and Forsyth used virtual reality simulation as a project of computerized teaching strategy in a university nursing school to develop students' clinical thinking [47]. Through the virtual reality simulation practice of venous catheter insertion, it can reduce the anxiety of teachers and students about the safety of patients and trial and error in real patients and students' anxiety. There are also many research studies that apply virtual reality technology to desktop virtual system software to cultivate students' clinical thinking ability. This kind of software emphasizes that the scene and the patient's discomfort reaction are displayed through the computer screen and the operator is immersed in the virtual situation. According to the relevant data and information, the purpose of nursing for patients' discomfort and pain is to train students to exercise appropriate and scientific problem-solving ability according to the patient's condition in complex situations [48, 49].

### 4.3. Virtual Reality Technology Promotes the Cultivation of Clinical Thinking of Medical Students

#### 4.3.1. Virtual Reality Technology Promotes the Development of Clinical Reasoning for Medical Students

Wang et al. compared the effect of immersion (experimental group) and nonimmersion (control group) virtual reality technology in intravenous injection experimental teaching under the trinity of “real person training + model assistance + virtual training.” The results show that virtual reality technology can effectively improve the clinical reasoning ability of learners [50]. Molina Carmona et al. proposed to train students to use targeted learning activities based on virtual reality applications and evaluate the improvement of students' spatial perception ability through widely accepted spatial visualization tests. It is found that virtual reality technology can promote the development of learners' visual spatial ability [51]. There is a strong correlation between the score of high-level visual spatial test and hand movement efficiency of novice surgeons. By testing spatial perception, such as orientation, visualization, and kinesthetic imagination, we found that spatial perception can affect clinical decision-making and clinical performance; for example, visuospatial ability can affect the clinical manifestations of periodontal plastic surgery [52]. Spatial perception can promote clinical decision-making and affect the performance of laparoscopic navigation task in the virtual learning environment [53].

#### 4.3.2. Virtual Reality Technology Promotes the Development of Critical Thinking in Medical Students

In the virtual reality learning environment, learners can interact with the objects in the virtual environment and get more intuitive perceptual objects. In the process of operation, they unconsciously take the initiative to think and stimulate their thinking process of finding, analyzing, and solving problems. Teachers encourage learners to reflect seriously, which is conducive to the cultivation of students' critical thinking ability [54]. Faridi et al. believe that virtual reality can effectively provide better visualization effect, and interaction with real 3D virtual reality can simplify the object of learning experience. An experimental study was carried out to determine that virtual reality intervention has a significant positive impact on students' learning and critical thinking [55]. Virtual reality technology can promote the interaction between learners, environment, and learning content. Previous studies have shown that interaction can promote the development of deeper learning and critical thinking. The development of clinical thinking is inseparable from the interaction between learners, learning content, patients, teachers, and environment. Rich technical tools and learning resources provide the foundation and support for the development of critical thinking. The richness of technical tools and resources brings convenience for the interaction between students and students, and between students and learning resources. The smoothness of communication also has an impact on the development of collective and individual higher-order thinking [56].

## 5. Conclusions

Virtual reality technology provides a realistic clinical learning environment for medical students, which can avoid risks, allow trial and error, and have repeatability and reversibility. In this paper, through the deconstruction of clinical thinking, this study determined the connotation and elements of clinical thinking, including clinical reasoning, clinical judgment, decision-making, and critical thinking. This paper discusses the influence of virtual reality technology on the development of clinical thinking, clinical reasoning, and critical thinking of medical students. Virtual reality technology can effectively promote the development of learners' visual spatial ability, and spatial perception ability can affect clinical decision-making and clinical performance. It can not only effectively provide better visualization effect but also make learners interact better with the environment and learning content, which can promote the development of deeper learning and critical thinking. This paper only theoretically analyzes the impact of virtual reality technology on medical students' clinical thinking, and the next work is to carry out empirical research on the basis of theoretical research.

## Figures and Tables

**Figure 1:** Elements of clinical thinking.

**Figure 2:** Model framework of virtual reality technology promoting the development of clinical thinking in medicine.

**Table 1:** Virtual reality technology promotes the cultivation of clinical thinking of medical students.

Virtual reality	Cultivation of clinical thinking
Immersion and interaction	They provide experience support for the cultivation of clinical thinking of medical students
Immersion and imagination	They provide visual spatial perception support for the cultivation of clinical thinking of medical students

## Data Availability

The data used to support the findings of this study are available from the corresponding author upon reasonable request.

## References

[1] Opinions of the Ministry of Education (2018). The national health commission and the state administration of traditional Chinese medicine on strengthening the cooperation of medical education and implementing the excellent doctor education and cultivation plan 2.0. *Bulletin of the Ministry of Education of the People’s Republic of China*.

[2] Zhou J., Xu C., Li P. (2020). Logical direction and innovative practice of medical humanities education under the background of “new medicine”. *Chinese Journal of Medical Education Research*.

[3] Gao P. (2020). Exploration on “excellent doctor cultivation plan 2.0” of five-year clinical medicine-taking the practice of excellent doctor cultivation in Xinxiang medical college as an example. *Chinese Health Service Management*.

[4] He K., Wang L. (2019). Development strategy of “new medicine” under the background of healthy China. *Chinese Journal of Engineering Science*.

[5] Tan J., Luo J., Tang S., Chen Z. (2020). Research status and hotspots of virtual reality technology in medical education–visualization analysis of knowledge map based on CNKI. *China Medical Education Technology*.

[6] Fu H., Xiong Y., Chen H., Liu H., Zhao H. (2017). Application status and thinking of VR technology in clinical medicine. *China Medical Education Technology*.

[7] Peng S. (2020). The idea and action of new medicine. *Journal of Shanghai Jiaotong University*.

[8] Shen R., Wang Y. (2020). Research on the logic, problems and action path of “new medicine” construction. *Medicine & Philosophy*.

[9] Zhang Y., Guo M., Du H., Su J., Fu X., Jiang X. (2015). Deepening the integration of basic medical courses and strengthening the cultivation of clinical thinking. *China Higher Medical Education*.

[10] Guo J., Yin zuojuan, Sui S. (2010). Analysis on the current situation of clinical thinking training of nursing staff. *Journal of Nursing*.

[11] Chen W., Guo J., Chen J., Xu P. (2010). Problems and analysis of clinical thinking training of medical students. *Modern Hospital*.

[12] Lim F. A. (2011). Questioning a teaching strategy to foster clinical thinking and reasoning. *Nurse Educator*.

[13] Sun Y., Feng S., Zhao X., Wang G. (2020). Analysis on the effect of self-developed VR teaching software for clinical practice ability training. *China Continuing Medical Education*.

[14] Zhao Y., Jing L., Chen C., Zhang P., Li S. (2015). Application of virtual reality technology in experimental teaching of nursing specialty. *Nursing Research*.

[15] Bordage G., Grant J., Marsden P. (2010). Quantitative assessment of diagnostic ability. *Medical Education*.

[16] Likhterman L. B., Kravchuk A. D., Okhlopkov V. A., Éliava S. S., Iakovlev S. B. (2014). Clinical thinking of a neurosurgeon. *Voprosy neirokhirurgii imeni N.N. Burdenko*.

[17] Chris D. M., Jenny D., Paul G. (2006). *Clinical Thinking, Evidence, Communication, and Decision-Making*.

[18] Fuks A., Boudreau J. D., Cassell E. J. (2009). Teaching clinical thinking to first-year medical students. *Medical Teacher*.

[19] Wang C. (2001). Clinical thinking training of medical students. *Journal of Fujian Medical University (Social Science Edition)*.

[20] Zeng Y., Lu Y. (2005). On the concept of clinical thinking. *Chinese Journal of Medical Education Research*.

[21] Faucher C. (2011). Differentiating the elements of clinical thinking. *Optometric Education*.

[22] Luis P. G. (2012). Description of clinical thinking by the dual-process theory. *Revista Medica de Chile*.

[23] Takata Y., Stein G. H., Endo K. (2013). Content analysis of medical students’ seminars: a unique method of analyzing clinical thinking. *BMC Medical Education*.

[24] Neistadt M. E. (1987). Classroom as clinic: a model for teaching clinical reasoning in occupational therapy education. *American Journal of Occupational Therapy*.

[25] Elstein A. S., Shulman L. S., Sprafka S. A. (1978). *Medical Problem Solving: an Analysis of Clinical Reasoning*.

[26] Jiang Y., Yuan X., Zuo X., Huang Y. (2021). Application of clinical thinking teaching in the teaching of medical undergraduate diagnosis. *Chinese Journal of Diagnostics*.

[27] Lin D. F., Xin A., Li J. A. (2020). Training of clinical diagnosis thinking in symptomatology theory teaching. *Chinese Journal of Diagnostics*.

[28] Sittig D. F., Wright A., Osheroff J. A. (2008). Grand challenges in clinical decision support. *Journal of Biomedical Informatics*.

[29] Huang L., Lu J., Liang Y., Huang Y., Zhao X. (2015). Correlation between critical thinking ability and general self-efficacy of medical students. *Fudan Education Forum*.

[30] Jiang Y. (2017). *Research on the Construction of Higher Order Thinking Development Model in Technology Rich Classroom Environment*.

[31] Lin C. (2005). Cultivating thinking quality is the breakthrough to develop intelligence. *Journal of National Academy of Education Administration*.

[32] Linden L. L. (2008). The effect of clinical simulation and traditional teaching versus traditional teaching alone on critical thinking of nursing students.

[33] Jing L., Gao J., Jia Y., Wang K. (2019). Development and application of virtual experiment project of nursing clinical thinking training. *Studies in Health Technology and Informatics*.

[34] Jauhiainen V. S., Pulkkinen D. (2009). Problem-based learning and e-learning methods in clinical practice. *Studies in Health Technology and Informatics*.

[35] Cowen V. S., Kaufman D., Schoenherr L. (2016). A review of creative and expressive writing as a pedagogical tool in medical education. *Medical Education*.

[36] Cai H. (2020). The connection of behaviorism, connectionism and symbolism. *Journal of Shanxi Normal University (Philosophy and Social Sciences edition)*.

[37] Zheng Y. (2015). Exploration on the teaching mode of College Students’ personalized learning from the perspective of Neo constructivism. *The Journal of Distance Education*.

[38] Wang M., Zheng X. (2015). Embodied cognition and learning environment: a theoretical review from the perspective of educational technology. *Open Education Research*.

[39] Wang C. (2020). Substitution and Transcendence of virtual teaching aids for physical teaching aids: from the perspective of embodied cognition. *E-Education Research*.

[40] Wang C. (2018). The theory of embodied cognition: situational interaction supported by technology. *E-Education Research*.

[41] Gao Y., Liu D. J., Huang Z. Z., Huang R. H. (2016). The core elements and challenges of virtual reality technology to promote learning. *China Educational Technology*.

[42] Shi S. (2020). Realistic representation and essential attribute of virtual learning style. *Contemporary Educational Science*.

[43] Zheng S., Li Y., Ye X. (2019). Deep learning in medical ultrasound analysis: a review. *Computer Engineering and Applications*.

[44] Liu S., Wang Yi, Yang X. (2019). Application of deep learning in medical ultrasound image analysis. *Engineering Times*.

[45] Duan M., Zheng H. (2021). Research on the model of advanced thinking training based on deep learning. *Modern Educational Technology*.

[46] Li C. E., Li D. M. (2019). Construction of deep learning model based on virtual reality environment. *CIN: Computers, Informatics, Nursing*.

[47] Jenson C. E., Forsyth D. M. (2012). Virtual reality simulation: using three-dimensional technology to teach nursing students. *CIN: Computers, Informatics, Nursing*.

[48] Mendez K. J. W., Piasecki R. J., Hudson K. (2020). Virtual and agumended reality: implication for the feature on nursing education. *Nurse Education Today*.

[49] Wang J., Xi W., Dong L. (2020). Application and challenge of virtual simulation technology in nursing education. *Chinese Journal of Nursing Education*.

[50] Wang P., Yan W., Wang F., Wang L., Cai H., Chen W. (2020). Application of immersive virtual reality technology in experimental teaching of intravenous injection method. *Chinese Nursing Management*.

[51] Molina Carmona K. R., Luisa Pertegal-Felices S. J., Jimeno-Morenilla M. F., Anastakis D. J., Grober E. D., Reznick R. K. (2018). Virtual reality learning activities for multimedia students to enhance spatial ability. *Sustainability*.

[52] Wanzel R., Hamstra C., Caminiti D., Demartines N., Gantert W. A. (2003). Visual-spatial ability correlates with efficiency of hand motion and successful surgical performance. *Surgery*.

[53] Rosenthal R., Hamel C., Oertli D., Demartines N., Gantert W. (2010). Performance on a virtual reality angled laparoscope task correlates with spatial ability of trainees. *Indian Journal of Surgery*.

[54] Tan H., Luo N., Tang A., Singh G., Gargrish S. (2020). Research status and hotspots of virtual reality technology in medical education-visualization analysis of knowledge map based on CNKI. *China Medical Education Technology*.

[55] Faridi H., Tuli N., Mantri A., Gurjinder S., Shubham G. (2020). A framework utilizing augmented reality to improve critical thinking ability and learning gain of the students in Physics. *Computer Applications in Engineering Education*.

[56] Nie S. (2017). *Research on Influencing Factors of College Students’ Critical Thinking Development in Online Learning Environment*.

